# *In Vivo* Efficacy, Toxicity Assessment, and Elemental Analysis of Traditionally Used Polyherbal Recipe for Diarrhea

**DOI:** 10.1155/2022/5977795

**Published:** 2022-08-22

**Authors:** Sakina Mussarat, Muhammad Adnan, Shaheen Begum, Alamgeer, Riaz Ullah, Alicja Kowalczyk

**Affiliations:** ^1^Department of Botany, Kohat University of Science and Technology, Kohat 26000, Khyber Pakhtunkhwa, Pakistan; ^2^Department of Environmental Sciences, Fatima Jinnah Women University, Rawalpindi, Pakistan; ^3^College of Pharmacy, University of Punjab, Lahore, Pakistan; ^4^Department of Pharmacognosy, College of Pharmacy, King Saud University, Riyadh, Saudi Arabia; ^5^Department of Environmental Hygiene and Animal Welfare, Wrocław University of Environmental and Life Sciences, Chełmońskiego 38C, Wrocław 51-630, Poland

## Abstract

A polyherbal formulation consisting of *Mentha piperita* L., *Camellia sinensis* L. Kuntze, and *Elettaria cardamomum* (L.) Maton with a ratio of 10 : 5 : 2, respectively, was recommended for curing nausea, vomiting, and diarrhea. Experimental validation is crucial to affirm its therapeutic property leads toward the development of modified antidiarrheal agents. This research aimed to investigate the *in vivo* antidiarrheal efficacy of traditionally used polyherbal recipe in a castor oil-induced animal model. Moreover, the study also presents the elemental screening and *in vivo* toxicity of tested polyherbal recipe. Individual plant parts of the polyherbal recipe were mixed according to the traditional prescription ratio, and hydromethanolic extract was prepared by the cold maceration process. The antidiarrheal activity was assessed by castor oil induction method, charcoal meal test, and enteropooling procedure in Sprague-Dawley rats. Elemental analysis and *in vivo* subacute toxicity were carried out, followed by biochemical, hematological, and histopathological analyses. Polyherbal extract significantly delayed the diarrhea onset in a dose-dependent manner and showed marked inhibition at 200 and 400 mg/kg. Fecal weight was reduced significantly (*p* < 0.05) at 200 mg/kg (0.26 ± 0.25) in comparison with the control (1.63 ± 0.15). The diarrhea score was zero at a concentration of 200 and 400 mg/kg. Antienteropooling effect of the extract was greater than that of loperamide. Following subacute toxicity, all the treated rats were normal, survived, and showed no changes in behavior. There were no significant differences between values of blood parameters in both the control and extract-treated groups except a significant decrease in monocytes (control 8.4; polyherbal 2.2). Elemental analysis showed a slight increase in the amount of manganese (Mn, 8.076 ppm) as compared to the WHO recommended level (2 ppm). Traditionally used polyherbal recipe is effective and safe for combating diarrheal diseases. *In vivo* evidence supported the use, safety, and efficacy of the polyherbal recipe that has been used as an alternative medicine for diarrhea in the study area. Inhibition of castor oil-induced diarrhea and antisecretory effect of the studied polyherbal recipe makes it a potent antidiarrheal drug without no or limited toxic effects at the tested dose after further analysis.

## 1. Introduction

Gastrointestinal disorders, including diarrhea, constipation, and stomach problems, remain a burden on human health, and most of these problems develop due to an imbalance of defensive and aggressive factors. Diarrhea is characterized by frequently loose bowel movements with increased liquid in the stool [1]. It is the second leading cause of mortality, accounting for 1 in 9 deaths in children, about 76,000 children suffering from diarrhea, and 1.7 billion cases per year [2]. Acute diarrhea is mainly caused by enteric pathogens like *Vibrio cholerae*, *Escherichia coli*, *Shigella,* and *Salmonella* species and some fungal and viral agents [3]. A previous study [4] indicates that 19% of 259 diarrheal patients have *Pseudomonas aeruginosa* as a causative agent. Oral rehydration solution, use of antibiotics, and antisecretory drugs are frequently used to cure diarrhea globally. Although oral rehydration therapy is effective in more than 90% of cases of dehydration due to diarrhea, it is ineffective in shortening the duration and stool frequency [5]. On the other hand, antibiotics and antisecretory drugs induce side effects as well as a chance of drug resistance development in microorganisms and disrupt the normal microbiota of the gastrointestinal tract. Consequently, there always remains a challenge for researchers to formulate new and alternate modes of treatment for curing diarrhea on urgent bases.

Complementary and alternative medicines in the form of plants earned the attention of people for curing different diseases due to their fewer side effects and easy access. Up to 2007, one-half of all registered drugs were derived from natural products or their derivatives, and about 122 compounds, which are currently part of allopathic medicines, are derived from ethnomedicinal plant resources, resulting in a remarkable surge in herbal medicine. Ethnomedicinally, various medicinal plants with antidiarrheal efficacy are widely used by local people and scientifically proven for diarrheal treatment [6–10], but still, there remains a challenge for the scientific community to explore the nature to produce more effective medicines. Nowadays, along with monotherapy, there is an increasing trend towards polytherapy to minimize the antibiotic resistance issue. Polyherbal therapy includes herbs-herbs combination as well herbs-antibiotics combination. Although the biological properties of most individual plants have been previously documented, however, their combination may show enhanced activity and synergistic effects that are less explored [11–13]. Decoction of three plants (*Mentha piperita L*. (leaves), *Camellia sinensis L*. (leaves), and *Elettaria cardamomum* (L.) Maton (fruit), with a ratio of 10 : 5 : 2) was used traditionally and considered very effective in treating diarrhea, nausea, and vomiting by people of the southern regions of Khyber Pakhtunkhwa [14]. This polyherbal mixture has a good inhibition zone against diarrhea, causing bacterial and fungal pathogens [15]. There is no study reported previously for its validation on a scientific basis, so this study was planned to investigate the curative and preventive effect of the traditionally used polyherbal combination against castor oil-induced diarrhea in an animal model and to test the toxic and effective dose through *in vivo* subacute toxicity. Moreover, the presence of essential and toxic elements was analyzed in the selected polyherbal recipe.

## 2. Materials and Methods

### 2.1. Data Collection and Selection of Polyherbal Recipe

The selected polyherbal recipe was commonly used by the local communities of Dera Ismail Khan, Khyber Pakhtunkhwa, Pakistan [14]. Oral and written consent was taken from participants who used this polyherbal mixture, locally named “*Podeena Qehwa*,” for digestive problems, including diarrhea. Moreover, the selected polyherbal recipe significantly inhibited the growth of bacterial pathogens [15]. Plant species comprising this mixture were identified at the Department of Botany, Kohat University of Science and Technology, Kohat, and submitted to the herbarium. Taxonomic identification, correction, and synonym of the collected plant species used in traditional polyherbal medicine were authenticated using the international plant name index (http://www.ipni.org), the plant list (http://www.theplantlist.org), and the flora of Pakistan (http://www.efloras.org).

### 2.2. Preparation of Polyherbal Extract

Collected plants used in the polyherbal recipe were washed, cut into small pieces, shade dried, and crushed into powder form with the help of a grinder. The powder of individual plants was mixed according to the traditional description for the polyherbal mixture (Table 1).

The powder of 100 g polyherbal mixture was drenched in 1000 ml of 80% methanol in a 2000 ml flask and kept for 7–15 days for allowing total extraction at room temperature by the cold maceration process. After that, the soaked polyherbal mixture was filtered by Whatman filter paper no. 41. The filtrate was collected in a beaker and evaporated through a rotary evaporator. The semisolid extract was preserved for experimental purposes.

### 2.3. Ethical Approval

This study was approved by the Research Ethical Committee of Kohat University of Science and Technology, Kohat, Ref. No. 17–12/2017.

### 2.4. Antidiarrheal Activity

#### 2.4.1. Animals Grouping and Dosing

Sprague–Dawley rats (180–200 g; either sex) housed at the Animal Resources Center, University of Sargodha, were used in this study. Rats were kept for one week in the experimental environment supplied with food and water ad libitum. The rats were maintained and handled according to the guideline of the National Institutes of Health (NIH). All administrations were done via the oral route, and the maximum volume administered was 2 ml. Following grouping, rats were abstained from feeding for 18–24 hours and were placed in an individual cage underlined with a white plastic sheet.

#### 2.4.2. Castor Oil-Induced Diarrhea Model

Fifteen rats were abstained from food for 18 hours with water ad libitum and divided into five groups having three animals each. Group 1 served as negative control administered with normal saline (10 ml/kg body weight), and group 2 served as positive control administered with loperamide (5 mg/kg body weight). Groups 3, 4, and 5 received polyherbal hydromethanolic extract in doses of 100, 200, and 400 mg/kg body weight, respectively, [8, 16]. After 30 min, 1.5 ml of castor oil was given to all experimental rats, they were kept in respective metabolic cages, and feces were collected. Rats were observed for 4 h, and diarrheal droppings were collected and weighed. A numerical score (solid: 0, semisolid: 1, and diarrhea: 2) was assigned to stool consistency and severity of diarrhea compared with control [17]. Total numbers of dry and wet stools were determined, and percent inhibition of defecation (PI Def) and diarrhea (PI Di) was calculated as follows:

  PI Def = mean number of feces (negative control − polyherbal or drug-treated group) / mean number of feces in negative control × 100.
  PI Di = mean number of diarrheal feces (negative control − polyherbal treated group) / mean number of diarrheal feces in negative control × 100).

#### 2.4.3. Castor Oil-Induced Enteropooling

Inhibition of fluid accumulation in the intestine by the tested polyherbal extract was measured by the method of [18]. Fifteen mice abstained from food for 18 hours with water ad libitum, and rats were grouped as above in the castor oil-induced method. After one hour of castor oil administration and polyherbal extract, rats were slaughtered, and the small intestine from the pylorus to the caecum was dissected and weighed. The intestinal content of each treated rat was collected, volume was measured, and the empty intestine was reweighed. Then, percent reductions in the weight of intestinal content (PR in Wt.) and volume of intestinal content (PR in Vol.), relative to the control group, were calculated as follows:

    PR in Wt. = Wt. of intestinal content (g) (negative control − polyherbal treated group) / Wt. of intestinal content (g) in the negative control × 100.
  PR in Vol. = Vol. of intestinal content (ml) (negative control − polyherbal treated group) / Vol. of intestinal content (ml) in the negative control × 100.

#### 2.4.4. Gastrointestinal Motility Test

Fifteen overnight fasted rats with free access to water were grouped as above, containing three animals in each group. After one-hour administration of polyherbal extract and castor oil, half ml of 5% charcoal suspension was given orally to measure the distance traveled. After a half hour, all rats were slaughtered, the small intestine of each mouse was dissected from pylorus to caecum, distance traversed by charcoal marker was measured, and percent inhibition (PI) of intestinal transit was calculated as follows [19]: PI of intestinal transit = % intestinal transit of charcoal marker (negative control − polyherbal treated group) / % intestinal transit of charcoal marker in the negative control × 100.

#### 2.4.5. *In Vivo* Antidiarrheal Index

*In vivo* antidiarrheal index (ADI) was calculated by a formula developed in [19]:

(1) $$\begin{array}{c} \text{ADI}=3\sqrt{D\text{ freq}\times G\text{ meq}\times P\text{ freq}}, \end{array}$$

where *D* freq is the delay in diarrhea onset, *G* meq is the reduction in charcoal distance, and *P* freq is the inhibition in diarrhea (%age).

### 2.5. Subacute Oral Toxicity

For the safety assessment of the effective dose of polyherbal crude extract, the subacute oral toxicity method was followed [20,21]. Distilled water was given orally to the control group (*n* = 5/group). Polyherbal mixture was dissolved in distilled water that was used as a vehicle. Polyherbal mixture was given orally to the second group according to body weight by oral gavage daily after 24 hr for 14 days. All the rats were closely observed for any change in their physical behavior within the first 30 min, then for 4 hours, and then subsequently for 14 days [22]. On the last day of the study, all animals were weighed and humanely sacrificed, and blood samples were collected in ethylenediaminetetraacetic acid (EDTA) tubes for biochemical (urea, creatinine, bilirubin, alanine aminotransferase (ALT), and alkaline phosphate (ALP)) and hematological (hemoglobin (Hb), RBC, platelet count, neutrophils (N), lymphocytes (L), monocytes (M), mean corpuscular hemoglobin (MCH), and mean corpuscular hemoglobin concentration (MCHC)) analyses. Vital organs such as kidneys and liver were removed and preserved in 10% formalin for histopathological examination. Prepared slides were studied under a light microscope; magnified images of tissues were captured for further study.

### 2.6. Elemental Detection

For elemental analysis, the polyherbal material was acid digested following standard procedure [23]. Briefly, the polyherbal materials were shade dried at room temperature and then in an oven at 60–80°C for 1 hr. In 10 mL concentrated HNO_3_, 1 g of manually crushed polyherbal sample was dissolved and then digested for 24 hours in a 50 mL calibrated test tube. On a Technicon block digester (Model BD-40), the sample was slowly heated to prevent excessive frothing. The temperature was raised gradually to 210°C to reduce the volume of HNO_3_ to 5 mL. After cooling, 2 mL of 72% HClO_4_ was added, and the heating was maintained for 0.5 hr until white HCIO_4_ vapors emerged in the test tube. The cooled sample was diluted up to 50 mL using distilled water. Dilution resulted in the formation of white precipitate, which was dissolved by warming the sample with hot water (75–80°C) [23].

Elemental analyses of Pb, Mn, Ni, Cu, Cr, Fe, Cd, Ca, K, Mg, Na, and Co were carried out in the selected polyherbal recipe by using a flame atomic absorption spectrophotometer (FAAS), Hitachi Ltd., 180–50. S. N5721, UV spectrometer for Na, and flame photometer for K, at Fatima Jinnah Women University Rawalpindi. For each element, a suitable working standard solution was drawn. Concentration versus absorbance calibration curves was developed. The data were statistically examined by using the fitting of a straight line. During the calculation of various elements, a blank reading was also taken, and any necessary corrections were performed.

### 2.7. Data Analysis

*In vivo* antidiarrheal results represent the mean and standard error, and the effect of the polyherbal extract was statistically compared with standard drug or normal saline group using ANOVA single factor analysis and *t*-test in Microsoft Excel 2007. *P* ≤ 0.05 was taken as statistically significant.

## 3. Results

### 3.1. Antidiarrheal Activity

#### 3.1.1. Polyherbal Extract Reduced Castor Oil-Induced Diarrhea

After 4 hours of observations, all the rats in the control group (normal saline 10 ml/kg, p.o.) produced copious watery diarrhea due to the administration of castor oil. The polyherbal extract-treated groups and standard drug loperamide (5 mg/kg) showed a significant delay in the onset of diarrhea and stool frequency. The polyherbal extract showed significantly delayed diarrhea onset in a dose-dependent manner; however, it showed marked inhibition at 200 and 400 mg/kg, and there were no diarrheal feces passed by any rats. The polyherbal extract also decreased the number of defecation times, but the comparison was nonsignificant. No stool was passed by any rats at a dose level of 400 mg/kg of polyherbal hydromethanolic extract which showed 100% inhibition of defecation or they might be constipated.

The weight of stool at a concentration of 200 mg/kg was 0.26 ± 0.25 (*P* < 0.05) and reduced significantly in comparison with the normal saline group (1.63 ± 0.15) (Table 2). The severity of diarrhea was significantly reduced, and the diarrhea score was zero at 200 and 400 mg/kg extract concentration (Table 3).

#### 3.1.2. Antienteropooling Effect of Polyherbal Extract

Intestinal fluid quantity generated by castor oil induction evaluated by enteropooling assay leads toward preventive measurements. Significant reductions in mean weights of the intestinal contents were 0.8 ± 0.34 (100 mg/Kg), 0.53 ± 0.20 (200 mg/kg), and 0.16 ± 0.05 (400 mg/kg), while the mean volumes of the intestinal content were 1.1 ± 0.26, 0.73 ± 0.25, and 0.36 ± 0.11 ml, respectively. The percent inhibition in volume was 60.14, 73.55, and 86.95%, and weight was 58.54, 72.53, and 91.7% at three tested doses, respectively, which was greater than standard drug (Figure 1).

#### 3.1.3. Effect on the Intestinal Transit of Charcoal Meal in Rats

The polyherbal extract significantly inhibited the movement of charcoal meal in castor oil-induced rats from the pylorus to caecum in a dose-dependent manner (100 and 200 mg/kg (*p* < 0.05) and 400 mg/kg (*p* < 0.01)) in comparison with negative control. The tested dose of 400 mg/kg also produced a significant effect (*p* < 0.05) in comparison with the standard drug loperamide. A higher significant reduction was observed in % intestinal transit of charcoal meal in a dose-dependent manner (100 mg/kg (50.64 ± 1.1), 200 mg/kg (30.04 ± 1.38), and 400 mg/kg (25.48 ± 2.81)). The tested dose of 400 mg/kg produced a statistically highly significant (*p* < 0.05) reduction when compared with the standard drug loperamide (43.98 ± 2.12). Compared to the negative control group receiving distill water, percent suppression in intestinal transit is 24.48%, 54.66%, 62%, and 34.41% at three doses of polyherbal extract and loperamide 5 mg/kg, respectively (Figure 2).

#### 3.1.4. *In Vivo* Antidiarrheal Index

*In vivo* antidiarrheal index (ADI) was used to check the antidiarrheal effect of the tested drug by using values in the formula. The polyherbal extract showed an antidiarrheal index of 74.42 (100 mg/kg), 110.15 (200 mg/kg), and 114.87 (400 mg/kg) at the three tested doses and indicated a dose-dependent effect on the ADI value (Table 4).

### 3.2. Elemental Analysis

Elemental analysis showed that no lead (Pb) was detected in the polyherbal extract, while the concentration of iron (Fe) was high (21.078 ppm) but within the permissible limit of the WHO (2007). The concentration of manganese (Mn) exceeded the permissible limit set by the WHO (2007). The concentration of chromium (Cr), cadmium (Cd), nickel (Ni), and cobalt (Co) was noted to be within the permissible limit of the WHO (2007) (Figure 3).

### 3.3. Subacute Toxicity

#### 3.3.1. Effects on the Behavioral Pattern and Body Weight

There was no sign of any toxicity and mortality after 14 days of receiving a 400 mg/kg dose of polyherbal extract regularly. No significant abnormal changes were observed in the liver, kidney, heart, and other vital organs of tested rats. There was no change in the physical behavior of polyherbal-treated rats compared to the control rats (Table 5). There was a gradual increase in the body weight of both control and polyherbal-treated rats for 1st week of the study, but in the 2nd week, there was a slight decrease in the body weight of the extract-treated rats without any significant difference (*p > 0.05*) (Figure 4). On 1st day of the study, control rats had a mean body weight of 133.6 ± 15.3, and on the final day, it was 136.8 ± 14.2, while the mean body weight of polyherbal treated rats was 166 ± 4.1, and the final mean body weight was 143.2 ± 15.5.

#### 3.3.2. Effects on Hematological and Biochemical Parameters

In the subacute study, hematological parameters, such as hemoglobin (Hb), total RBC, platelet count, and lymphocytes (*L*), and biochemical parameters of the polyherbal extract-treated group at 400 mg/kg concentration were within the normal range and were not significantly different from the control (Table 6). There was a significant decrease in the percentage of monocytes (*M*) compared with the control (2.2 ± 1;*p* < 0.05).

#### 3.3.3. Effects on Histology of the Liver and Kidneys

Histopathology of liver and kidney sections treated with both normal saline (control rats) and polyherbal extract (400 mg/kg) treated rats showed a normal appearance of endothelial cells and veins. There were no microscopic changes shown compared with the control. There were no necrosis and hemorrhage seen in polyherbal crude extract-treated rats (Figure 5).

## 4. Discussion

Traditional herbal formulations have been used as alternative medicine by different herbal industries and local practitioners for treating many diseases, including gastrointestinal complaints [13, 24, 25]. In this study, a traditionally used polyherbal formulation for diarrhea was tested on an animal model. There is scarce data available for polyherbal combinations used by local people providing an experimental base, so there is a need to justify the commonly used polyherbal combination through *in vivo* trial. Traditionally used polyherbal recipe consists of three plants: *Mentha piperita* (Leaves), *Camellia sinensis* (Leaves), and *Elettaria cardamomum* (Fruit) with a 10 : 5 : 2 ratio. The antimicrobial potential of these individual plants was well documented in the literature [26–28]. Published literature of a five-year period regarding antimicrobial research and plant synergy concludes that synergy both within plant extract and between plants and antibiotics can give more efficient antimicrobials than isolated constituents [29]. The studied polyherbal formulation has an inhibitory effect on common bacterial pathogens [15]. Extraction of the polyherbal formulation through 80% methanol may have a potent antimicrobial effect due to the presence of biologically active ingredients, as hydromethanol has the ability to dissolve both polarities. Due to the aquaphobic property of essential oils present in *M. piperita* and *E. cardamomum*, they split lipids of the cell membrane and mitochondria, making them permeable, causing a leak of cell contents, and leading to cell death of bacteria [30].

Administration of castor oil significantly induced diarrhea in rats after 69.66 ± 7.23 min. Castor oil has a laxative effect due to the presence of ricinoleic acid and is widely used for the comparison of antidiarrheal screening of test drugs. Castro oil reduces fluid absorption and increases electrolyte secretion because the compound responsible causes irritation of intestinal mucosa that enhances the secretion of endogenous prostaglandins, nitric oxide, platelet-activating factor, tachykinins, and cAMP intracellular accumulation [3]. Polyherbal recipe reduced the number of feces and 100% inhibition of diarrhea. The weight of stools (0.26 ± 0.25) and severity of diarrhea are significantly reduced (*P* < 0.05) as compared to control, and the diarrhea score is zero at 200 and 400 mg/concentration. The inhibitory effect of this formulation may be due to the blockage of all the intracellular accumulation promoted by castor oil. Results in this study are similar to those in previous studies [16, 31], where the dose-dependent antidiarrheal effect was produced by a single plant. The antidiarrheal effect of the polyherbal mixture may be due to some active constituents that inhibit intestinal secretion and induce a relaxing effect on smooth muscles. Flavonoids, polyphenols, and tannins reported from individual plants present in this polyherbal formulation may produce a relaxant effect on smooth muscle, alternately inhibiting diarrhea.

Polyherbal mixture showed a significantly higher antisecretory effect of intestinal accumulation, even more than standard drug. This may be due to an increase in the ability of water reabsorbing capacity and smooth muscle relaxation. Nonsteroidal anti-inflammatory drugs can suppress castor oil-induced diarrhea. Similarly, *E. cardamomum* showed an anti-inflammatory effect in a previously reported study [32]. Osmotic and/or secretory mechanisms are disturbed in diarrhea, alternatively affecting the absorption-secretion process. SGLT1 transporter maintains the absorption pathway, increasing the reabsorption of fluids during diarrhea when ORT therapy starts [33]. Published literature reported that terpenoids and steroids like phytosterols could suppress the production of prostaglandin E2 [34], a stimulating hormone of intestinal secretions. Reduction in intestinal motility is another way to inhibit symptomatic diarrhea. Loperamide interacts with intestinal opioid receptors, inhibits gastrointestinal transit, and increases reabsorption [35]. The polyherbal extract produced a significant reduction in charcoal movement in the intestine. Charcoal is a nonabsorbable agent used as a marker for distance traveled through the intestine. The highest percent inhibition in intestinal transit was 62% at 400 mg/kg, which is greater than the standard drug (34.41%), suggesting that there are some factors involved in the reduction of intestinal motility. The parasympathetic nervous system releases acetylcholine that plays an important role in regulating bowel movements by promoting contraction of the smooth muscle. By inhibition of this neurotransmitter, intestinal transit can be slow [36]. Possible anticholinergic effects of the combination of plants are recommended for further studies.

The presence of metal concentrations and their complexation with chemotherapeutic agents influence the efficacy of medicinal plants in curing various diseases. These metals are involved in the formulation of active chemical components and are hence responsible for both therapeutic and harmful qualities [37]. The standardization of the dosage of herbal medicines can be determined after analyzing the essential and toxic elements in them. Therefore, it is important to determine the level of these metals in herbal medicine as, at elevated levels, they may exert adverse effects. The WHO/FAO has proposed the limit of concentrations in the medicinal and edible fruit plants. The permissible limit for Cr in plants is 0.02 ppm, set by the FAO/WHO [38], while according to the WHO (2007), it is 1 ppm. In this study, the polyherbal extract met the reference range set by the WHO (2007) and FAO/WHO [38]. The allowed limit of Pb in medicinal plants is 10 ppm [39]. Pb is considered the most hazardous environmental pollutant which accumulates in the bones, causes behavioral abnormalities, acts as a neurotoxin, and retards intelligence and mental growth [40]. The permissible limit for Mn in plants is 2 ppm, set by the FAO/WHO [38]. In comparison to the present data, the polyherbal mixture accumulated Mn and crossed the permissible limit. In literature, a high intake of Mn produces adverse effects on the function of the brain, lungs, and central nervous system (CNS) [41, 42]. Copper, as a micronutrient, has critical biological functions, but higher concentrations could be toxic [43]. In the studied polyherbal mixture, Cu concentration was lower than the permissible limit set by the FAO/WHO (3 ppm). The polyherbal recipe showed Cd concentrations in line with 0.3 ppm recommended for medicinal plants by the WHO [38]. In contrast to the present results, excessive accumulation of Cd in plants in urban areas of Peshawar can be related to various anthropogenic activities [44].

All the treated rats were normal, survived, and showed no change in behavior with no significant difference in biochemical and hematological parameters. Behavioral and physiological changes are due to certain enzymes regulated by aspartate transaminase (AST) and alanine transaminase (ALT). Polyherbal extract-treated rats have no significant change in the level of AST and ALP, which alternately has no effect on mood swings. Urea and creatinine, which regulate renal function, were in the normal range with that of control, and histopathological examination of kidneys showed normal architecture. So, the tested dose was nontoxic and effective in diarrhea inhibition.

## 5. Conclusions

Results revealed that natural flora plays a vital role in the primary healthcare of people and is helpful in eliminating acute infectious and chronic diseases. It is supposed from the results that the polyherbal recipe consists of several compounds that may act synergistically to produce the desired therapeutic effects, which may be lost by individual usage. Present evidence affirms the therapeutic efficaciousness and safety of this polyherbal formulation for treating diarrhea. There is no toxic element exceeding the prescribed limit in the evaluated recipe. However, further research is needed to identify the active compounds responsible for the antidiarrheal effect and mechanism of action. Toxicity study shows that an effective dose for inhibiting diarrhea is also nontoxic and does not cause any toxic signs in tested animals. Hence, the tested polyherbal remedy is further recommended for phytochemical and biological invesitgation.

## Figures and Tables

**Figure 1:** Antienteropooling effect of the polyherbal extract in albino rats. (a) Inhibition in the volume of intestinal content. (b) % inhibition in the volume of intestinal content. (c) Inhibitory effect on the weight of intestinal content. (d) % inhibition in the weight of intestinal content. Values are represented as mean ± standard error (*n* = 3); ^*∗*^*P* < 0.01; ^∗∗^*P* < 0.001 compared with the negative control.

**Figure 2:** Effect of polyherbal extract on intestinal transit in albino rats. (a) Effect on intestinal transit. (b) % intestinal transit. (c) % inhibition of intestinal transit. Values represented as mean ± SEM (*n* = 3); ^*∗*^*p* < 0.05; ^∗∗^*P* < 0.01 compared with the negative control.

**Figure 3:** Elemental analysis of polyherbal recipe.

**Figure 4:** Effect of polyherbal extract on body weight (g) of albino rats at concentration 400 mg/kg.

**Figure 5:** Histopathological study of liver and kidney. (a) Liver of normal control rat showing normal architecture. (b) Liver of polyherbal extract-treated rat without any effect on tissues. (c) Kidney of normal control rat showing normal architecture. (d) Kidney of polyherbal extract-treated rat without any damage to tissue.

**Table 1:** Individual plants of polyherbal recipe (*Podeena Qehwa*).

Individual plant botanical name/voucher no/family/local name/English name/part used/quantity	Disease treated
*Mentha piperita* L./KUH-353a/Labiatae/Podeena/mint/leaves/10 g	Decoction (tea) is used for nausea, vomiting, and diarrhea
*Camellia sinensis* (L.) Kuntze/KUH-464/Theaceae/Sabz chaey/green tea/leaves/5 g	
*Elettaria cardamomum* (L.) Maton/KUH- 487/Zingiberaceae/Sabz illaichi/green cardamom/fruit/2 g	

**Table 2:** Effect of polyherbal recipe extracts on castor oil-induced diarrhea.

Groups	Onset of diarrhea (min)	No. of diarrheal feces	Inhibition of diarrhea %	Total no. of feces	Inhibition of defecation %	Total weight of feces	Rats with diarrhea	% rats protected
Control (normal saline + co)	69.66 ± 7.23	8.66 ± 0.57	—	8.66 ± 0.57	—	1.63 ± 0.15	3	0
Loperamide 5 mg/kg + co	211 ± 4.58^∗∗∗^	0.66 ± 0.57	92.37	4.99 ± 2.07	42.37	0.70 ± 0.1^∗∗^	1	66.66
Recipe 100 mg/kg + co	196.66 ± 75.05	0.66 ± 0.57	92.37	1.99 ± 0.63	77.02	1.16 ± 0.85^*∗*^	1	66.66
Recipe 200 mg/kg + co	240 ± 0^∗∗∗^	0	100	0.66 ± 0.51	92.37	0.26 ± 0.25^*∗*^	0	100
Recipe 400 mg/kg + co	240 ± 0^∗∗∗^	0	100	0	100	0^∗∗^	0	100

Values taken as mean ± SEM (*n* = 3), one-way ANOVA. ^∗∗^ = *P* < 0.01, ^∗∗∗^ = *P* < 0.0001, and ns = nonsignificant versus control.

**Table 3:** Castor oil-induced diarrhea score for polyherbal recipe.

Treatment group	Watery feces × 2	Semisolid × 1	Solid × 0	Cumulative score
Control	6.60	2.20	0.0	15.10 ± 1.16
Loperamide 5 mg/kg	0.00	0.60	4.60	0.60 ± 0.40^*∗*^
Recipe (100 mg)	2	2	2	6 ± 2
Recipe (200 mg)	0	0	2	0^∗∗^
Recipe (400 mg)	0	0	0	0^∗∗^

Values taken as mean ± SEM (*n* = 3), one-way ANOVA. ^∗∗^ = *P* < 0.01, ^∗∗∗^ = *P* < 0.0001, and ns = nonsignificant versus control.

**Table 4:** *In vivo* antidiarrheal index (ADI).

Treatment group	Delay in diarrhea onset (*D* freq %)	Peristaltic index %	*G* meq %	Purging frequency	*P* freq %	ADI
Control	—	67.06 ± 3.68	—	8.66 ± 0.57	—	—
Loperamide 5 mg/kg	202.89	43.98 ± 2.12	34.41	0.66 ± 0.57	92.37	86.39
Recipe (100 mg)	182.31	50.64 ± 1.10	24.48	0.66 ± 0.57	92.37	74.42
Recipe (200 mg)	244.53	30.40 ± 1.38	54.66	0	100	110.15
Recipe (400 mg)	244.53	25.48 ± 2.81	62	0	100	114.87

**Table 5:** Physical patterns of albino rats in polyherbal crude extract-treated (400 mg/kg) and control groups.

Parameters	Observations											
	30 minutes		4 h		24 h		48 h		7 days		14 days	
	CG	PG	CG	PG	CG	PG	CG	PG	CG	PG	CG	PG
Skin appearance	√	√	√	√	√	√	√	√	√	√	√	√
Eyes	√	√	√	√	√	√	√	√	√	√	√	√
Mucous membrane	√	√	√	√	√	√	√	√	√	√	√	√
Respiratory system	√	√	√	√	√	√	√	√	√	√	√	√
CNS	√	√	√	√	√	√	√	√	√	√	√	√
Somatomotor activity	√	√	√	√	√	√	√	√	√	√	√	√
Behavioral pattern	√	√	√	√	√	√	√	√	√	√	√	√
Sleep	√	√	√	√	√	√	√	√	√	√	√	√
Coma and convulsion	Nf	Nf	Nf	Nf	Nf	Nf	Nf	Nf	Nf	Nf	Nf	Nf
Salivation	√	√	√	√	√	√	√	√	√	√	√	√
Lethargy	Nf	Nf	Nf	Nf	Nf	Nf	Nf	Nf	Nf	Nf	Nf	Nf
Urination (color)	√	√	√	√	√	√	√	√	√	√	√	√
Itching	Nf	Nf	Nf	Nf	Nf	Nf	Nf	Nf	Nf	Nf	Nf	Nf
Feces consistency	√	√	√	√	√	√	√	√	√	√	√	√
Mortality	Nf	Nf	Nf	Nf	Nf	Nf	Nf	Nf	Nf	Nf	Nf	Nf

CG = vehicle control group, PG = polyherbal extract-treated group, √ = normal and good, and Nf = not found.

**Table 6:** Effect of polyherbal crude extract and vehicle treatment on blood parameters.

Parameter index		Unit	Normal saline group	Polyherbal group
Biochemical parameters	Blood urea	mg/dl	71.4 ± 11	62.8 ± 5.8
	Serum creatinine	mg/dl	1.24 ± 0.1	1.08 ± 0.1
	S bilirubin	mg/dl	0.7 ± 0	0.8 ± 0
	ALT	U/L	64.2 ± 8.9	58.6 ± 36.5
	ALP	U/L	513 ± 236.4	310.2 ± 94

Hematological parameters	Hb	g/dl	10.96 ± 0.7	10.94 ± 0.9
	RBC count	10^*∗*^6/ul	5.21 ± 0.4	5.50 ± 0.5
	TLC	10^*∗*^3/ul	3.40 ± 1	5.45 ± 2.8
	Lymphocytes	%	52 ± 4	53.8 ± 21.5
	Neutrophils	%	38 ± 1.4	38.2 ± 22.7
	Monocyte	%	8.4 ± 4.1	2.2 ± 1^*∗*^
	Platelets	10^*∗*^3/ul	605.6 ± 125.7	486.2 ± 309
	MCV	fL	56.8 ± 0.61	55.8 ± 0.63
	MCHC	g/dl	33.06 ± 0.3	33.4 ± 0.56

Values represented as mean ± SEM, *n* = 5.

## Data Availability

All the available data are incorporated into the paper.
